The article "Learning Generative State Space Models for Active Inference" was published in 2020. Journal: Front Comput Neurosci.

# Learning Generative State Space Models for Active Inference

**DOI:** 10.3389/fncom.2020.574372

**Published:** 2020-11-16

**Authors:** Ozan Çatal, Samuel Wauthier, Cedric De Boom, Tim Verbelen, Bart Dhoedt

**Affiliations:** IDLab, Department of Information Technology, Ghent University - imec, Ghent, Belgium

**Keywords:** active inference, free energy, deep learning, generative modeling, robotics

## Abstract

In this paper we investigate the active inference framework as a means to enable autonomous behavior in artificial agents. Active inference is a theoretical framework underpinning the way organisms act and observe in the real world. In active inference, agents act in order to minimize their so called free energy, or prediction error. Besides being biologically plausible, active inference has been shown to solve hard exploration problems in various simulated environments. However, these simulations typically require handcrafting a generative model for the agent. Therefore we propose to use recent advances in deep artificial neural networks to learn generative state space models from scratch, using only observation-action sequences. This way we are able to scale active inference to new and challenging problem domains, whilst still building on the theoretical backing of the free energy principle. We validate our approach on the mountain car problem to illustrate that our learnt models can indeed trade-off instrumental value and ambiguity. Furthermore, we show that generative models can also be learnt using high-dimensional pixel observations, both in the OpenAI Gym car racing environment and a real-world robotic navigation task. Finally we show that active inference based policies are an order of magnitude more sample efficient than Deep Q Networks on RL tasks.

## 1. Introduction

Enabling intelligent behavior in artificial agents has been one of the long standing goals of the machine learning community (Russell and Norvig, 2009). Historically this has been tackled in various different ways, starting from logic agents and knowledge bases and evolving into complex neural network based reinforcement learning (RL) methods. Artificial intelligence agents have made incredible progress in the field of game playing. Ranging from beating the world chess champion in 1997 (King, 1997) to beating the world Go champion in 2016 (Silver et al., 2017).

Major advances in autonomous behavior are driven by deep neural networks on the one hand and the application thereof in reinforcement learning on the other hand. In RL, agents optimize their policy by interacting with an environment in order to maximize a scalar reward signal. Despite recent advances in solving games with reinforcement learning (RL), this leap in intelligence however has not manifested itself as much in real world cases, such as robotics (Irpan, 2018). This is caused by a number of limitations of the current RL methods. First, RL algorithms typically do not perform as well in the real world due to their notoriously bad sample efficiency (Kurenkov, 2018). In order to learn, agents need to perform a lot of (bad) interactions to improve their policy. Second, to be able to start improving a policy, RL agents first need to find at least some reward. Sometimes it is sufficient to introduce some random exploration, but often a more complex exploration strategy is required, using concepts such as novelty or curiosity (Abbeel and Ng, 2005). Third, whereas games have an obvious and well-defined reward definition such as a score or the ability to win the game, it is much harder to define and obtain a consistent and relevant reward signal for a real-world task (Wiewiora, 2010). Finally, RL agents are generally trained with a single task in mind. Generalizing to new tasks either requires retraining or fine-tuning the agent, or requires the addition of meta-learning components (Hospedales et al., 2020).

The article "Learning Generative State Space Models for Active Inference" was published in 2020. Journal: Front Comput Neurosci.

Human beings on the other hand grow up and learn new tasks without the need for an external reward signal (Oudeyer and Kaplan, 2007). A promising emerging theory from cognitive neuroscience, called active inference, provides a mathematical framework rooted in physical and biological observations describing the mechanisms of natural agency and behavior in the human brain (Dayan et al., 1995; Rao and Ballard, 1999; Friston, 2010).

Active inference rests upon the free energy principle for the brain (Friston, 2010), which models the brain as a Bayesian inference engine. The free energy principle states that every self-organizing system in environmental equilibrium must be minimizing its free energy (Friston et al., 2006). Free energy in this respect can be seen as a proxy for “surprise” or prediction error, and offers a unified account of action, perception and learning (Friston, 2010). The free energy principle has been able to explain a wide array of anatomical and physiological aspects of brain systems (Angelucci et al., 2002; Bastos et al., 2012; Friston et al., 2017a) Furthermore it allows for an elegant treatment of the intricate relationship between perception and action while inherently balancing the exploration and exploitation trade-off.

In recent years, active inference has been demonstrated in a lot of use cases, ranging from decision making under uncertainty to structure learning, navigation, etc., an overview is given in Da Costa et al. (2020). In these cases an agent is typically equipped with a predefined, discrete state space generative model of its environment, on which the agent performs inference and learning. Although such simulations showcase the effects of active inference on the behavior of the agent studied, this is impractical for applications in the real-world, where it is impossible to engineer such a generative model. However, we know that natural selection can learn such models in a biological setting. This means, in principle, it is possible to learn a generative models of the world. In what follows, we show that this is the case using deep learning. Recently there has been an increase in research on the application of deep learning to active inference (Ueltzhöffer, 2018; Tschantz et al., 2019; Millidge, 2020). However, these approaches either specify some parts of the state space beforehand or only treat low dimensional observations.

The article "Learning Generative State Space Models for Active Inference" was published in 2020. Journal: Front Comput Neurosci.

In this paper, we use recent advances in deep neural networks to learn generative models of the world purely from experienced action-observation pairs without specifying any part of the agent state space. We show that agents equipped with these models can engage in active inference by free energy minimization while achieving high sample efficiency. We demonstrate our approach on three use cases with increasing complexity: the mountain car problem (section 3.1), the OpenAI Gym car racing environment (section 3.2), and a real-world robot navigation task (section 3.3). We benchmark our approach against DQN, a well-known RL baseline, and show that our approach is able to achieve significantly higher rewards in a low-data regime.

## 2. Methods

### 2.1. Active Inference

Any agent, either artificial or natural, can only perceive the surrounding environment (characterized by its hidden state *h*) through sensory observations, and changes its environment through actions. The implicit sensory blanket (Figure 1) separates external (environmental) states from the internal states of an agent –that entail a generative model of the external states. An agent's action at time step *t* will change the environment's *hidden* state ***h***_*t*_ according to some generative process $R\left(\tilde{o},\tilde{a},\tilde{h}\right)$ over sequences of observations $\tilde{o}$, actions $\tilde{a}$ and hidden states $\tilde{s}$; and provide new observations ***o***_*t*_ to the agent. We will use tildes to designate sequences in the remainder of this paper. However, as the agent has no direct access to the hidden states of the environment, it can only develop its own internal belief states ***s***_*t*_ that explain the perceived observations as well as possible, by means of a generative model.

The article "Learning Generative State Space Models for Active Inference" was published in 2020. Journal: Front Comput Neurosci.

**Figure 1:** An agent's Markov blanket. An agent has no direct access to the environment's hidden states $\tilde{h}$. It can only perceive the consequences of its actions ***a***_*t*_ by means of observations ***o***_*t*_, and develop its own internal belief states ***s***_*t*_. Note that ***s***_*t*_ does not necessarily have to match the environments hidden states ***h***_*t*_. Tildes indicate sequences of observations, actions or hidden states.

More concretely, the agent's world model can be formalized as partially observable Markov decision process (POMDP), with the probability distribution $P\left(\tilde{o},\tilde{s},\tilde{a},\pi \right)$, specifying the joint probability of the agent's observations, belief states, actions and policies. In this formalism a policy is nothing more than a sequence of actions *a*_*t*:*T*_ up until some time horizon *T*. Without loss of generality, we assume the world model is Markovian, so that the agent's state ***s***_*t*_ at time step *t* is only influenced by the previous state ***s***_*t*−1_ and action ***a***_*t*−1_. Graphically this model can be visualized through time according to Figure 2A. Formally, it can be factorized as follows:

(1) $$\begin{array}{l} P\left(\tilde{o},\tilde{s},\tilde{a},\pi \right)=P\left(s_{0}\right)P\left(\pi \right)\overset{T}{\underset{t=1}{\prod }}P\left(o_{t}|s_{t}\right)P\left(s_{t}|s_{t-1},a_{t-1}\right)P\left(a_{t-1}|\pi \right). \end{array}$$

**Figure 2:** **(A)** The POMDP depicting an agent's model of the world up until the current timestep *t*. The current state *s*_*t*_ determines the current observation ***o***_*t*_ and is only influenced by the previous state ***s***_*t*−1_ and action ***a***_*t*−1_. Both actions and observations are assumed to be observed, indicated by a gray coloring, whereas states need to be inferred. **(B)** The agent's model of the world from timestep *t* onward. As with the model for the past we assume that for each timestep the observation is only influenced by the corresponding state. Note that for the future we assume the agent has control over which states to visit through its actions which are determined by a policy π.

Due to the separation between the agent and the environment through the Markov blanket, the agent is only able to infer the effects of its actions on the world through observations. This entails that the agent can only update its beliefs over world states through Bayesian inference on possible belief state values conditioned on observed actions and observations. In fact the agent tries to infer its belief state value ***s*** through the posterior belief $P\left(\tilde{s}|\tilde{o},\tilde{a}\right)$. The actual posterior in this form, derived directly from Bayes rule is, in general, intractable to calculate directly from the given joint model in Equation (1). To avoid this, the agent resorts to variational inference (Beal, 2003), and approximates the true posterior by some approximate posterior distribution $Q\left(\tilde{s}|\tilde{o},\tilde{a}\right)$, which is in a form that is tractable to the agent. Similar to the model posited in Equation (1), the approximate posterior distribution can be decomposed as:

(2) $$\begin{array}{l} Q\left(\tilde{s}|\tilde{o},\tilde{a}\right)=Q\left(s_{0}|o_{0}\right)\overset{T}{\underset{t=1}{\prod }}Q\left(s_{t}|s_{t-1},a_{t-1},o_{t}\right). \end{array}$$

In active inference, the agent is believed to be acting according to the free energy principle, which states that every agent's goal is to minimize its variational free energy. In view of our generative model, the variational free energy *F* is formalized as (Friston, 2013):

(3) $$\begin{array}{l} F={𝔼}_{Q(\tilde{s}\text{|}\tilde{o},\tilde{a})}\left[\log Q\left(\tilde{s}\text{|}\tilde{o},\tilde{a}\right)-\log P\left(\tilde{o},\tilde{s},\tilde{a}\right)\right]\\ \;=\underset{posterior\;approximation}{\underset{︸}{D_{KL}\left[Q(\tilde{s}\text{|}\tilde{o},\tilde{a})||P(\tilde{s}\text{|}\tilde{o},\tilde{a})\right]}}-\underset{log\;evidence}{\underset{︸}{\log P(\tilde{o})}}\\ \;=\underset{complexity}{\underset{︸}{D_{KL}\left[Q\left(\tilde{s}\text{|}\tilde{o},\tilde{a}\right)||P\left(\tilde{s},\tilde{a}\right)\right]}}-\underset{accuracy}{\underset{︸}{{𝔼}_{Q(\tilde{s}\text{|}\tilde{o},\tilde{a})}\left[\log P(\tilde{o}|\tilde{s})\right]}}. \end{array}$$

When rewriting the variational free energy using the second equality, it decomposes into two terms: the KL-divergence between the approximate and true posterior distribution, and the (negative) log evidence. This means that minimizing free energy is equivalent to maximizing the log evidence, while making the posterior approximation as good as possible. One can also see that the variational free energy is actually the negative evidence lower bound, which is maximized in variational inference (Bishop, 2006). Variational free energy can also be written as the third equality, which comprises a complexity and accuracy term. This states that the model should minimize the complexity of accurate explanations of the observations (Schwartenbeck et al., 2019).

The article "Learning Generative State Space Models for Active Inference" was published in 2020. Journal: Front Comput Neurosci.

Note the omission of π in Equation (3), as we assume the agent has a (perfect) proprioceptive feedback channel, i.e., all executed actions are observed. For time steps in the future this is not the case, and the agent will have to make inferences about which policy (and actions) to select.

The crucial aspect of active inference is that agents not only try to minimize their free energy for past observations, but also aim to minimize their free energy in the future. For future time steps, the actions are determined by a chosen policy π, and both actions and observations are no longer observed, but become random variables that have to be inferred, as shown in Figure 2B. In order to minimize the free energy in the future, the agent not only needs to form posterior beliefs over its current state, but also form beliefs over future states and observations when following certain policies. This allows the agent to evaluate the so-called expected free energy *G* for some policy π, and form a belief over possible policies *P*(π) (Schwartenbeck et al., 2019) as:

(4) $$\begin{array}{l} P\left(\pi \right)=\sigma \left(-\gamma G\left(\pi \right)\right). \end{array}$$

This means the agent picks or samples policies according to some softmax σ function with temperature γ over the total expected free energy. Policies that exhibit low total expected free energy will have a higher likelihood to be sampled. The above equations denote a crucial aspect of active inference, namely that the only self-consistent prior belief over policies *P*(π) is to believe that the agent will follow policies that minimize the expected free energy (Friston K. et al., 2015).

The expected free energy is defined as the sum of the expected free energy of a policy over all timesteps that we look ahead in the future:

(5) $$\begin{array}{l} G\left(\pi \right)=\underset{\tau }{\sum }G\left(\pi ,\tau \right), \end{array}$$

with

(6) $$\begin{array}{l} \begin{array}{l} G\left(\pi ,\tau \right)={𝔼}_{Q\left(o_{\tau },s_{\tau }|\pi \right)}[\log Q\left(s_{\tau }|\pi \right)-\log P\left(o_{\tau },s_{\tau }|\pi \right)]\\ \;={𝔼}_{Q\left(o_{\tau },s_{\tau }|\pi \right)}[\log Q\left(s_{\tau }|\pi \right)\\ \;-\log P\left(o_{\tau }|s_{\tau },\pi \right)-\log P\left(s_{\tau }|\pi \right)]\\ \;=\underset{\text{risk}}{\underset{︸}{D_{KL}[Q\left(s_{\tau }|\pi \right)||P\left(s_{\tau }\right)]}}+\underset{\text{ambiguity}}{\underset{︸}{{𝔼}_{Q\left(s_{\tau }\right)}[H\left(P\left(o_{\tau }|s_{\tau }\right)\right)]}} \end{array} \end{array}$$

Note that we set *P*(***s***_τ_|π) = *P*(***s***_τ_), which reflects that the agent has a prior preference over which states to visit (Friston K. et al., 2015). One can interpret this as the agent having prior beliefs over states that it will visit, independent of a policy, but driving policy selection to these attractor states. An obvious example of a preferred state is for example maintaining a temperature of 37 °C (Van De Laar and De Vries, 2019). These preferred states basically determine the agent, and can be endowed on the agent either by nature through evolution, in the case of natural agents, or by humans in the case of artificial agents.

The article "Learning Generative State Space Models for Active Inference" was published in 2020. Journal: Front Comput Neurosci.

Two important parts emerge from Equation (6): the KL-divergence between the approximate posterior distribution over future states and their corresponding prior belief, called the risk, and the expected entropy over future observations, also known as the ambiguity (Friston et al., 2016). These terms illustrate the way an active inference agent will act. On the one hand the agent will try to match the states it visits in the future with its prior belief over future states, hence realizing preferences or exhibiting goal-directed behavior (Schwartenbeck et al., 2019). On the other hand the agent will try to reduce the conditional entropy on future observations, or avoid ambiguous states.

### 2.2. Active Inference and Deep Neural Networks

Current active inference schemes usually start by specifying the belief state space manually, in terms of a generative model. Variational Bayes is then used to infer hidden states and parameters under this model (Friston et al., 2009; Sajid et al., 2019; Van De Laar and De Vries, 2019). This approach works well for low-dimensional problems or problems where a sensible belief state can be devised for the task at hand. If the problem domain at hand is high-dimensional (e.g., the observations are in pixel space) or the dynamics are difficult to model manually (e.g., pedestrian dynamics for an autonomous car), it becomes exceedingly difficult to handcraft the agent's belief states. Instead, it would be better if the agent could *learn* its own representation and parameterization of the belief state space. To do so, we build and learn the generative model using deep artificial neural networks, which are trained on sequences of action-observation pairs.

#### 2.2.1. The Generative Model

To achieve state space learning, we map the different factors of the POMDP model of Equation (1) and the corresponding approximate posterior of Equation (2) to three neural network models: the transition model *p*_θ_, the likelihood model *p*_ξ_ and the posterior model *p*_ϕ_, as shown in Equation (7).

(7) $$\begin{array}{l} \begin{array}{l} P\left(\tilde{o},\tilde{s},\tilde{a}\right)=P\left(s_{0}\right)\overset{T}{\underset{t=1}{\prod }}\overset{p_{\theta }\left(s_{t}|s_{t-1},a_{t-1}\right)}{\overset{︷}{P\left(s_{t}|s_{t-1},a_{t-1}\right)}}\cdot \overset{T}{\underset{t=0}{\prod }}\overset{p_{\xi }\left(o_{t}|s_{t}\right)}{\overset{︷}{P\left(o_{t}|s_{t}\right)}}\\ Q\left(\tilde{s}|\tilde{o},\tilde{a}\right)=Q\left(s_{0}|o_{0}\right)\overset{T}{\underset{t=1}{\prod }}\underset{p_{\phi }\left(s_{t}|s_{t-1},a_{t-1},o_{t}\right)}{\underset{︸}{Q\left(s_{t}|s_{t-1},a_{t-1},o_{t}\right)}} \end{array} \end{array}$$

The transition model *p*_θ_ takes as input a previous state and action pair, and outputs a distribution of the current state. The approximate posterior model *p*_ϕ_ also outputs a distribution of the current state, but in addition to the previous state and action, also receives the current observation as input. Finally the likelihood model *p*_ξ_ outputs a distribution of the current observation, given the current state. The output distributions of these neural networks are each parameterized as a multivariate normal distribution with diagonal covariance matrix, i.e., each neural network outputs the means μ and standard deviations σ of N(μ,σ). Assuming a multivariate normal distribution of this kind can be regarded as restricting the class of generative models to the same distributional forms used in mean field approximations of the variational posterior. In other words, we make simplifying assumption that the generative model can itself be factorized by precluding off diagonal terms in the covariance matrix.

The article "Learning Generative State Space Models for Active Inference" was published in 2020. Journal: Front Comput Neurosci.

Rolling out through time is done in a recursive manner, as shown on Figure 3. At each time step *t*, a sample ***s***_*t*_ is drawn from the posterior state distribution, which is forwarded through the transition model and posterior model to get the next state distribution, and through the likelihood model to obtain an observation estimate. At *t* = 0 we start with the initial observation and a zero vector for the state and action.

**Figure 3:** The generative model is parameterized by 3 neural networks. The Transition Model models the prior probability of going from state ***s***_*t*−1_ to ***s***_*t*_ under action ***a***_*t*−1_. The Posterior models the same transition while also incorporating the current observation ***o***_*t*_. Finally the likelihood model decodes a state sample ***s***_*t*_ to a distribution over possible observations. These models are used recurrently, meaning they are reused every time step to generate new estimates.

#### 2.2.2. Training the Model

To optimize these neural network models we first obtain a dataset of sequences of action-observation pairs by interacting with the environment. This can for example be obtained using a random policy or by human demonstrations. We then train the models end-to-end on this dataset using stochastic gradient descent by minimizing the free energy loss function:

(8) $$\begin{array}{l} L=\underset{t}{\sum }D_{KL}[p_{\phi }\left(s_{t}|s_{t-1},a_{t-1},o_{t}\right)||p_{\theta }\left(s_{t}|s_{t-1},a_{t-1}\right)]-\log p_{\xi }\left(o_{t}|s_{t}\right) \end{array}$$

This resembles the loss function of a Variational Autoencoder (VAE) (Kingma and Welling, 2014; Rezende et al., 2014), in which the posterior model acts as the encoder and the likelihood model as the decoder. The loss then consists of a (negative) log likelihood term penalizing reconstruction errors, and a KL-divergence between the posterior and a prior distribution. However, in comparison with a VAE where typically a standard normal prior is used, in our case the prior for time step *t* is provided (and learned) by the transition model.

The article "Learning Generative State Space Models for Active Inference" was published in 2020. Journal: Front Comput Neurosci.

To allow the gradient flow through the sampling step, we use the reparameterization trick, by which samples of a multivariate Gaussian distribution parameterized by means ***μ*** and standard deviations ***σ*** are calculated as:

(9) $$\begin{array}{l} s=\mu +\epsilon ⊙\sigma ,\;\epsilon_{i}\sim N\left(0,1\right). \end{array}$$

Also note that we approximate the expectation of the accuracy term in Equation (3) by a single sample in the loss function. In practice this works due to the stochastic gradient descent procedure that operates on batches of data per optimization step.

#### 2.2.3. Planning as Inference

To engage in active inference using the trained models, we need to infer the empirical prior *P*(π) for each policy π. We start by generating imaginary rollouts from the learned transition model. The action trajectories used to generate different imaginary rollouts are then ranked according to expected free energy *G*. We then execute the first action of the policy (i.e., action sequence) π with the lowest *G*. By actually taking the action in the environment, the agent gets a new observation from the environment back. Which can then be used with the posterior model to generate a new starting state for the planning, after which the process outlined in this paragraph restarts.

Calculating the expected free energy *G* for all possible action sequence π requires calculating *G*(π, τ) using Equation (6), which involves estimating *Q*(***s***_τ_|π) and the expected entropy 𝔼*H*(*P*(***o***_τ_|***s***_τ_)). Our models however only consider a single time step at a time, so the only way to get estimates about future time steps τ is by iterative Monte Carlo sampling.

Concretely, for each policy π, we sample *N* state trajectories following π for *K* future time steps. As we have not yet observed future observations, we now sample from the transition model *p*_θ_ instead of the posterior model as ***s***_*t*+1 : *t*+*K*_ ~ *p*_θ_(·|***s***_*t*+1 : *t*+*K*−1_, π). This results in *N* state samples ${\hat{s}}_{\tau }$, for which we can sample *N* observation estimates ${\hat{o}}_{\tau }\sim p_{\xi }\left(\cdot |{\hat{s}}_{\tau }\right)$. To be able to calculate the KL-divergence we use a Gaussian distribution with parameters calculated from the sample batch means $\mu_{{\hat{s}}_{\tau }}$ and variances $\sigma_{{\hat{s}}_{\tau }}^{2}$. Similarly we use a Gaussian with mean $\mu_{{\hat{o}}_{\tau }}$ and variance $\sigma_{{\hat{o}}_{\tau }}^{2}$ to calculate the entropy. We can then estimate the expected free energy for each policy from current time step *t* onward as follows:

(10) $$\begin{array}{l} {\hat{G}}_{t}\left(\pi \right)=\overset{t+K}{\underset{\tau =t+1}{\sum }}D_{\text{KL}}[N\left(\mu_{{\hat{s}}_{\tau }},\sigma_{{\hat{s}}_{\tau }}\right)∥P\left(s_{\tau }\right)]+\frac{1}{\rho }H\left(N\left(\mu_{{\hat{o}}_{\tau }},\sigma_{{\hat{o}}_{\tau }}\right)\right)\\ \;+\underset{\pi^{\prime }}{\sum }\sigma \left(-\gamma {\hat{G}}_{t+K}\left(\pi^{\prime }\right)\right){\hat{G}}_{t+K}\left(\pi^{\prime }\right) \end{array}$$

The first summation term looks *K* timesteps ahead, calculating the KL-divergence between expected and preferred states and the entropy on the expected observations. We also introduce an additional hyperparameter ρ, which allows for a trade-off between reaching preferred states on the one hand and resolving uncertainty on the other hand. This hyperparameter can be regarded as nuancing the effective precision of prior preferences over states in the future. For example, a large value suppresses the contribution of the entropy term in the same way that increasing the precision of prior preferences would increase the contribution of the KL divergence or risk. In other words, ρ controls the risk aversion or greediness of the agent.

The article "Learning Generative State Space Models for Active Inference" was published in 2020. Journal: Front Comput Neurosci.

The second summation term implies that after *K* timesteps, we continue to select policies according to their expected free energy, hence recursively re-evaluating the expected free energy of each policy at timestep *t* + *K*. This allows us to limit the size of the search tree to multiples of *K* while still keeping in line with the theoretical grounds of the active inference framework. Calculation of *G* then unfolds as a search tree rooted at the current state estimate ***s***_*t*_, as shown in Figure 4. In fact, this scheduling scheme means that we run a particular action *K* times and then consider a switch in the action for *D* times. In practice, however, we evaluate the recursion *D* times, resulting in an effective planning horizon of *H* = *K* × *D*. We select a new action every time step, and then rebuild the search tree. This means that even though our policy search plans ahead with a fixed policy each *K* time steps, in reality we allow the agent to reevaluate and possibly switch its policy at every time step.

The article "Learning Generative State Space Models for Active Inference" was published in 2020. Journal: Front Comput Neurosci.

**Figure 4:** Estimating the expected free energy *G*(π) for each policy involves sampling state and observation trajectories using the transition and likelihood model. The depicted tree shows the first level of unfolding with *N* = 3 samples, *K* = 2 lookahead time steps and 2 policies π_1_, π_2_.

Note that in Equation (10), we replaced the expected conditional entropy in *E*_*Q*_*H*(***o***_τ_|***s***_τ_) by the unconditioned entropy *H*(***o***_τ_). As *H*(***o***_τ_) ≥ *H*(***o***_τ_|***s***_τ_) due to the elimination of the mutual information *I*(***o***_*t*_; ***s***_*t*_) (noting that the mutual information is always greater than zero), we effectively minimize is in fact an upper bound on the expected free energy.

## 3. Results

We evaluate our approach on three different problems of increasing complexity. We start with the continuous control mountain car problem, which has already been treated before in active inference literature (Friston et al., 2009) with a generative model specified upfront. Second, we address the OpenAI car racing problem, in which the agent has to keep a car on the road whilst only observing a low resolution topdown view of the car and the road. Finally, we train a model on a real world mobile robotics dataset and demonstrate the capacity of our model to imagine future outcomes of the world.

We aim to address the following research questions:

- Can the agent learn a generative model purely from data to engage in active inference?
- Does the generative model successfully capture the ambiguity in the environment?
- Does the agent exhibit goal-directed behavior by specifying a preferred state distribution?
- How does the agent compare to state of the art deep RL methods such as DQN?

### 3.1. Partially Observed Mountain Car

The mountain car problem is an often used reinforcement learning benchmark. It consists of a sinusoidal mountain range with the goal of driving an underactuated car on top of the taller mountainside. A rendering of the environment is found in Figure 5A. The simplicity of the environment allows us to know the ground truth world dynamics upfront. The agent state in the world ***h*** is defined as the position and velocity of the car as given by Moore (1990).

**Figure 5:** Description of the mountain car problem and model rollout results. **(A)** Shows a render from the environment with the position axis included. The car is shown at position −0.5 which is the starting position in our evaluations. The goal of the experiment is to drive an underactuated car up the right-hand mountainside. The only way to achieve this is to first go left to gain enough momentum. **(B)** Shows the posterior and prior reconstructions of a trained mountain car model on a rollout from a random agent over 300 timesteps. The transition model rollout is bootstrapped with the initial state value of the posterior model. Both prior and posterior believes follow the groundtruth accurately.

The article "Learning Generative State Space Models for Active Inference" was published in 2020. Journal: Front Comput Neurosci.

In spite of its apparent simplicity, this problem remains an interesting first benchmark for any dynamics modeling or behavior learning approach due to the sparseness of the reward, as the agent only receives reward when the car reaches the top of the hill. Also, the top can only be reached by first moving in the opposite direction to build up enough momentum to drive up the hill. As such, the mountain car problem is not solvable by greedy approaches that aim to directly move toward the mountain top.

In order to amend the mountain car to a POMDP formalism, we allow our agent to only observe a noisy estimate of its actual position and omit the velocity information. As to properly solve the resulting problem, the agent now has to learn how to model the velocity and denoised position in its belief state space ***s***. The agent can follow either policy π_*l*_ or π_*r*_, which each repeat the same action of either throttling to the left or the right. By switching between these policies at different time steps a more complex policy can be built. The low-dimensional nature of this problem allows us to explore the effect of the risk and ambiguity terms on *G*, and by extension on the learned behavior. Furthermore we experiment with two variants of the environment. The agent can start with a fixed zero initial velocity, or it can start with a randomized velocity. When starting with a randomized velocity the agent has to learn to quickly estimate its current velocity in order to estimate when to start driving right, increasing the problem complexity.

For our generative model, we instantiate *p*_θ_(***s***_*t*_|***s***_*t*−1_, ***a***_*t*_), *p*_ϕ_(***s***_*t*_|***s***_*t*−1_, ***a***_*t*_, ***o***_*t*_) and *p*_ξ_(***o***_*t*_|***s***_*t*_) as fully connected neural networks with two hidden layer containing 20 hidden neurons, and a 4-dimensional state space. The model architecture and parameterization were determined empirically. To bootstrap the model, we train on actions and observations of a random agent that randomly selects to throttle left or right with 10% chance, and repeats the previous action otherwise. The models are trained until convergence with a batch size of 32 sequences of length 100 each, minimizing the loss as described in Equation (8) using the Adam optimizer with learning rate 0.0001. We used PyTorch for the definition and training of all neural networks. The performance of the model is assessed through inspecting the difference between state reconstructions and ground truth values, illustrated in Figure 5B. Both the prior and posterior model are capable of estimating the ground truth observations accurately.

The article "Learning Generative State Space Models for Active Inference" was published in 2020. Journal: Front Comput Neurosci.

Next, we instantiate an active inference agent that uses Equation (10) to plan ahead and select the policy with the lowest expected free energy. As preferred state distribution *P*(***s***_τ_), we manually drive the car up the mountain and evaluate the model's posterior state at the end of the sequence ${\hat{s}}_{end}$, and set $P\left(s_{\tau }\right)=N\left({\hat{s}}_{end},1\right)$. To limit the computations, we allow the active inference agent to plan ahead for 90 timesteps, where policies are evaluated for *K* = 30 time steps, with a recursion depth of *D* = 3, and drawing *N* = 100 samples for each policy.

To evaluate the planning as inference, we visualize sampled trajectories for all branches of the search tree at *t* = 0, after observing only a single observation at start position −0.5. This is a challenging starting position as the car needs enough momentum in order to reach up the hill from there. In the case of a random starting velocity, the generative model is not sure about the velocity after only the first observation. This is reflected by the entropy (i.e., the expected ambiguity) of the sampled trajectories as illustrated in Figure 6. Now following π_*r*_ from the start will sometimes reach the preferred state, depending on the initial velocity. In this case the active inference agent's behavior is determined by the parameter ρ. For ρ>1, the agent will act greedily, preferring the policy that has a chance of reaching the top early, cf. Figure 6E. When setting ρ < <1, the entropy term will play a bigger role, and the agent will select the policy that is less uncertain about the outcomes, rendering a more cautious agent that prefers a more precise and careful policy, moving to the left first see Figure 6A. We found setting ρ = 0.1 yields a good trade-off between cautiousness and greediness for the mountain car agent.

**Figure 6:** We plot the agents imagined trajectories, in terms of imagined position, under different policies. Action sequences starting with a left action are colored red. Sequences starting with a right action are colored blue. Each action is repeated 30 times before picking a new action. Due to the random initial velocity, the car will reach the hill fast using the always right policy in only part of the samples **(E)**, however starting with the left policy first consistently reaches the hill top with low entropy on the observations **(A)**. A greedy agent (ρ > 1) will pick **(E)** whereas a cautious agent (ρ < < 1) will favor **(A)**. For each policy **(A–H)** we report the values of KL, H and G for ρ = 0.1.

The article "Learning Generative State Space Models for Active Inference" was published in 2020. Journal: Front Comput Neurosci.

In the environment with no initial velocity, the transition model learned by the agent is quite accurate and the entropy terms are an order of magnitude lower than the case with random initial velocity, as shown in Figure 7. However, in terms of preferred state the lowest KL-value is still achieved by following π_*r*_. This is due to the fact that the KL-term is evaluated each time step, and moving to the left, away from the preferred state in the sequence then outweighs the benefit of reaching the preferred state in the end. Choosing ρ = 0.1 again forces the agent to put more weight on resolving uncertainty, preferring the policy in Figure 7A.

**Figure 7:** As in Figure 6, we plot the agents imaginary trajectories for different policies. When the environment starts the car with a fixed zero velocity, the model is on average much more certain on the predicted trajectories, resulting in lower entropy terms. However, policy **(E)** still achieves the lowest KL value, as this term is evaluated each time step, and moving away from the preferred state yields a high KL penalty. When choosing ρ = 0.1, the agent again favors **(A)**. For each policy **(A–H)** we report the values of KL, H and G for ρ = 0.1.

We compare our approach with a often used reinforcement learning baseline for problems with discrete action spaces, DQN (Mnih et al., 2015). Similar to our active inference approach DQN learns from off-policy data, but however, it also explores the world with the policy it is learning. We compare the success rate of agents trained using active inference to DQN agents, trained on 10, 100, 1000 and 10 000 episodes. The DQN agents are parameterized by am MLP with two hidden layers of 200 neurons and are trained using stochastic gradient descent with a fixed ϵ value of 0.3, a γ of 0.99 and a learning rate of 0.001. We repeat the training process 10 times to account for effects of randomness on the training performance. Finally we repeat the evaluation run for each train run 100 times to eliminate the effects of randomness in the environment on the agents performance. In Figure 8A, we plot the average success rate and its spread for the active inference agents (orange) and the DQN agent (blue). Note that we did not train the active inference agent for 10,000 episodes as it already outperforms the DQN agent by a significant margin.

**Figure 8:** Comparison between DQN agents and Active Inference agents in terms of reward. We compare each agents performance when trained over 10, 100, 1,000, and 10,000 episodes. We trained each agent ten times for each episode amount to account for training instabilities. **(A)** Shows the success rate for both active inference agent (orange) and the DQN agent (blue) on the mountaincar problem. Note that success rate and reward are interchangeable here as an agent only gets a reward of one when reaching the top. We do not train the active inference agent for 10,000 episodes since it already consistently achieves a high success rate in 100 and 1,000 episodes. **(B)** Shows the reward score the car racing DQN agent (in blue) achieves. The Active inference agent is trained on only 10 episodes and is indicated in red.

The article "Learning Generative State Space Models for Active Inference" was published in 2020. Journal: Front Comput Neurosci.

If we zoom in on the active inference performance when only trained on a single rollout, we must note that the performance is very dependent on the content of the train data. Only if during this random sequence the car reaches the top, the agent is able to create a plan that solves the environment.

### 3.2. Car Racing

The aim of the car racing task is to keep a car on the road, observed from a top down 2D perspective as shown in Figure 9. The track is randomly generated every time the agent is reset. The action space comprises a vector indicating the steering angle, the amount of throttle and brake as continuous values, which we discretized to three possible policies: go forward, go left and go right. The observation space consists of RGB images of 96 by 96 pixels, as shown in Figure 9. The agents own internal state representation ***s*** is given by 16 independent Gaussian distributed state variables.

**Figure 9:** A render from the OpenAI gym car racing environment. The car will always be present in the bottom center of the image in this environment, the only parts that change in the observations will be the black bar at the bottom and the shape of the track.

We use the same general model architecture as in the mountain car experiments, instantiating *p*_θ_(***s***_*t*_|***s***_*t*−1_, ***a***_*t*−1_) as a multilayer perceptron with 128 hidden neurons. We use a VAE architecture for *p*_ξ_(***o***_*t*_|***s***_*t*_) and *p*_ϕ_(***s***_*t*_|***s***_*t*−1_, ***a***_*t*−1_, ***o***_*t*_). The conditioning on ***a***_*t*_ and ***s***_*t*−1_ is achieved by concatenating them to the feature vector generated by a convolutional pipeline on the initial input image *o*_*t*_. Details about the specific neural architecture can be found in Appendix A.

We have trained our models on a dataset consisting of seven human demonstration sequences on 7 tracks of varying length. We used the Adam optimizer with an initial learning rate of 0.0001 and a minibatch size of 32 consisting of subsequences of length 15. Due to the fact that the reconstructed observations are images where likelihood distributions are difficult to interpret, we fix the standard deviation of the resulting pixel likelihood distributions to 1. This in fact means that the negative log likelihood term in our loss function is equivalent to a mean squared error loss on the means of the likelihood distributions.

The article "Learning Generative State Space Models for Active Inference" was published in 2020. Journal: Front Comput Neurosci.

An example of model beliefs on a human rollout is given in Figure 10. The prior samples are generated from 10 samples out of the initial posterior distribution, and are only updated through the transition model using the previous state and action, resampling from the resulting prior distributions every timestep. The posterior samples are generated using the initial posterior state sample and then updating that sample using the posterior model from the previous state and action and the real observation. In Figure 10C, we see that the model is capable of modeling temporally coherent states from just previous beliefs and actions.

**Figure 10:** Visualization of the models belief states for a human rollout. Time flows from left to right. In **(A)**, we show the ground truth observations. In **(B)**, we show the reconstructions from a belief sample that was updated every time with both the real action and real observation. In **(C)**, we have the corresponding reconstructions from imagined belief states sampled by the transition model, after observing only the initial observation. As the position of the car is always fixed at the center bottom, the shape of the reconstructed road segments gives insight in how the agent performs.

Because the agent always starts at the middle of the road we take the initial frame of a rollout as preferred observation, which can be translated to a preferred state distribution $P\left(\tilde{s}\right)$ through the agents posterior model, as seen in Figure 11A. From this preferred state distribution and the trained model we then instantiate an active inference agent that uses Equation (10) in the same way as we did in the mountain car experiments, setting *K*, *D* and *N* to 10, 2 and 2, respectively. We also find that a ρ of 0.0001 yields the best results in terms of imaginary planning. This is possible due to the low variability in the environment and the environment lending itself to a greedy solution. We provide Figures 11B,C as references as how to interpret the expected entropy terms in this experiment. In these figures we overlay 10 different trajectories each starting from the same initial state with the same action sequence. If there is little variation in what the agent believes will happen, the imagined trajectories will overlap a lot, their superposition will become less blurry as can be seen in Figure 11B. However, if there is a lot of variation in the imaginary rollouts, the trajectories will overlap less, resulting in blurry images, as can be seen in Figure 11C. This visual blurriness correlates with the entropy of the planned trajectories.

The article "Learning Generative State Space Models for Active Inference" was published in 2020. Journal: Front Comput Neurosci.

**Figure 11:** **(A)** Shows the agents preferences generated from a human demonstration. The preferences specify that the agent should prefer to drive on the road instead of the grass. Note that here there is no temporal correlation between each frame in the sequence. **(B,C)** show how the expected entropy term of *G* can be interpreted in the case of our latent spaces. They show the superposition of 10 different imaginary trajectories under the same action sequence (forward, forward), with a look ahead of 2. Time flows from left to right in these sequences. The car is always in the bottom center of the image.

Finally it is worth noting that although the agents' preferences are defined only by situations with straight road segments, as seen in Figure 11A, the agent has no issues in driving through corners. Figure 12 shows the agent taking a sharp and straight corner, when the only option to safely navigate the corner is to keep on the road the agent will do just that (Figure 12A). However, when the corners are more shallow the agent will try to cut the corner in order to realize its preferences faster (Figure 12B).

**Figure 12:** Active inference agent performance in corners. The agent will sometimes cut shallow corners **(B)** in order to achieve its goals as fast as possible. When the corner is too sharp to safely cut **(A)** the agent will follow the road instead.

As with the mountaincar experiment, we benchmark our approach against DQN and compare the performance of a DQN agent trained for 10, 100, and 1,000 episodes against an active inference agent trained on only 10 episodes. We use the stable baselines3 (Raffin et al., 2019) implementation of DQN using the library's CNNPolicy. We train with stochastic gradient descent with a learning rate of 10^−4^ and a scheduled ϵ starting at 1 and decreasing linearly proportional with the training length up until a minimum of 0.05. The results are visualized in Figure 8B. As with the mountaincar setting, the active inference agent is able to obtain high rewards from a handful of demonstration rollouts, whereas a DQN agent requires a lot of interactions with the environment before it starts obtaining rewards.

### 3.3. Robotic Navigation

As a final experiment we test our technique on a robotics case. We collect a dataset of real world (camera image, action) pairs using a Kuka youbot (Figure 13) equipped with a Realsense RGB-D camera. Note that the depth information of the RGB-D camera is omitted.

The article "Learning Generative State Space Models for Active Inference" was published in 2020. Journal: Front Comput Neurosci.

**Figure 13:** The Robotic setup used to collect the real world data. The mobile platform is a Kuka Youbot, the data is captured with a Intel Realsense RGB-D camera.

We collect the data by driving the robot up and down the aisles of a warehouse lab. Action information is provided in the form of linear and angular velocity commands. All data is synchronized and recorded at a frequency of 10Hz. As can be seen in Figure 14, the added difficulty of this dataset is the amount of clutter that the real world offers in the observation space. Note as well, that in order to comprehend the effect of the action vector on the world effectively the model will also need to learn to translate its own velocity information to distortions and translations on the image feed in its belief space.

**Figure 14:** Experimental results: **(A)** Shows the target observation in imagined (reconstructed) space. **(B)** The start observation of the trial. **(C)** Shows different imaginary planning results, while **(D)** Shows the actually followed trajectory.

We use the same architecture as in the car racer experiment, keeping the VAE encoder and decoder networks, while changing *p*_θ_(***s***_*t*_|***s***_*t*−1_, ***a***_*t*−1_) to an LSTM to allow for more temporal depth in the prior transition model following the findings of Hafner et al. (2019). The exact parameterization of our models is provided in Appendix A. These models are trained with Adam optimizer using the objective function from Equation (8) for 1M iterations. We use a mini-batch size of 128 and a sequence length of 10 timesteps.

We utilize the same approach as in the mountain car and car racing problems for our imaginary trajectories and planning. The agent has access to three base policies to pick from: drive straight, turn left and turn right. Actions from these policies are propagated to the learned models at different time horizons *H* = 10, 25, or 55. For each resulting imaginary trajectory, the expected free energy *G* is calculated. Finally the trajectory with lowest *G* is picked, and the first action of the chosen policy is executed, after which the imaginary planning restarts. The robot's preferences are given by demonstration, using the state distribution of the robot while driving in the middle of the aisle. This should encourage the robot to navigate safely in the aisles.

At each trial the robot is placed at a random starting position and random orientation and tasked to navigate to the preferred position. Figure 14 presents a single experiment as an illustrative example. Figure 14A shows the reconstructed preferred observation from the given preferred state, while Figure 14B shows the trial's start state from an actual observation. Figure 14C shows the imagined results of either following the policy “always turn right,” “always go straight,” or “always turn left.” Figure 14D is the result of utilizing the planning method explained above.

The article "Learning Generative State Space Models for Active Inference" was published in 2020. Journal: Front Comput Neurosci.

The robot indeed turns and keeps driving in the middle of the aisle, until it reaches the end and then turns around^1^. When one perturbs the robot by pushing it, it will again recover and continue to the middle of the aisle due to the way the planning takes place in the agents belief space.

## 4. Discussion

We have shown in the above experiments that it is indeed possible to learn a generative active inference model purely from data without specifying any transition dynamics or meaning to the state spaces upfront. The required dataset size varies from problem domain to problem domain and can be collected by a random agent or human experts. We found that such a learned generative model can indeed capture the dynamics and the ambiguity of the environment well enough to be able successfully represent the environment in a its own belief states. From these belief states we can successfully plan ahead, giving rise to goal-directed behavior toward the preferred state distribution. Our approach is able to outperform DQN in terms of reward in a low-data regime without being trained specifically on solving the corresponding task. However, in order to achieve this sample efficiency, we assumed that the training data covers the real underlying distribution of observations and sufficiently covers the action space. This is the case for the problems on which we benchmarked, however for more complex environments the agent would need an improved and guided exploration mechanism. In addition, we currently train the generative model beforehand, and only afterwards we introduce the planning as inference. Ideally the agent should be trained while interacting with the environment, making the entire system end-to-end. This would require the agent to also evaluate expected free energy during the training process for exploration (Schwartenbeck et al., 2019), i.e., by maintaining a posterior distribution over model parameters similar to Tschantz et al. (2019).

One of the main difficulties in our approach of active inference is the specification of the preferred state distribution, as it generally requires that the corresponding preferred observation is already acquired in some way so that the desired state values can be calculated through the agents generative model. In the above experiments we acquired the desired observations either from the agents first observation (car racing experiment) or from human demonstration (mountain car and navigation experiment). However, as the generative model is trained, also this preferred state distribution can shift as the model can assign new meaning to state vectors trough the learning process. One way to mitigate this is by defining the preferences in terms of observations instead of states, as in Friston et al. (2016). However, this is impractical for high dimensional observations such as pixels. Another option is to embed a reward signal in the observation space as proposed by Tschantz et al. (2019), and put a prior preference on high reward outcomes.

The article "Learning Generative State Space Models for Active Inference" was published in 2020. Journal: Front Comput Neurosci.

Together with the specification of the preferred state distribution, one also determines how strong the agent is attracted by its preferences. For example, by defining the prior as a Gaussian distribution with low variance around a preferred state sample, the KL-term in Equation (6) becomes very large and overwhelms the ambiguity term. To overcome this issue we again make use of the ρ hyperparameter (Equation 10) which enables to weigh the two terms, resulting in a risk-taking or risk-averse agent, as shown in the mountain car experiment.

In our current experiments, we always trained the model on relatively short subsequences in comparison to the time horizon the agent needs to operate on. The downside of this, is that our model has a shallow temporal depth. The model cannot actually predict accurately far in the future, and also can not keep a mental “map” of the environment. In the robotic navigation experiment the model only knew that the aisles are straight and how to avoid obstacles. However, it could not differentiate between the different aisles. In the car racing experiment the model is also not able to predict entire circuits, it just knows that the road is a continuous object, and that after each segment it currently sees there will be another segment. Future work might focus on how to incorporate the current technique into hierarchical and temporally deeper models (Friston et al., 2017b), allowing the agent to reason on different levels of action abstractions.

Finally, in the current experiments we did not perform any pruning in the policy search tree, all possible branches of the tree were evaluated. This currently prevents the application of our approach to problems requiring significant temporal depth. However, as the expected free energy *G* is a non-negative additive quantity we could effectively prune the tree by eliminating all branches above a certain *G* value, following the principle of Occam's Window (Madigan and Raftery, 1994). Another path forward might be to replace the explicit planning by an amortized *habit* policy neural network which could be used in unsurprising states. The agent could then switch back to explicit, and expensive, planning when encountering uncommon, high surprise states.

The article "Learning Generative State Space Models for Active Inference" was published in 2020. Journal: Front Comput Neurosci.

### 4.1. Related Work

Active inference, as described by Friston since 2003 (Friston, 2003, 2010, 2013; Friston et al., 2006, 2009; Friston K. et al., 2015; Friston et al., 2016), has been applied to many different problem domains, highlighting the potential of a free energy driven artificial agent. Active inference based models have been shown to solve a wide array of tasks in different settings ranging from thermostats (Friston et al., 2012) to foraging problems (Mirza et al., 2016). In Friston et al. (2009, 2012), it is shown that a well-parameterized active inference model is capable of solving optimal control problems, including a discrete version of the mountain car problem. In Sajid et al. (2019), an in-depth comparison is made between active inference and reinforcement learning on the OpenAI Gym frozen lake environment. Other applications of active inference are text recognition (Friston K. J. et al., 2015), speech recognition (Kiebel et al., 2009a), perceptual categorization (Kiebel et al., 2009b), robotic arm control (Pio-Lopez et al., 2016). These approaches however all rely on a carefully specified generative model to operate successfully, a process that has to be done manually before any Bayesian inference on the model parameters proceeds. Our approach, on the other hand, leverages recent advances in the field of generative modeling (Higgins et al., 2017) using deep neural networks, allowing to fully learn a generative model from data.

A popular approach to generative modeling is variational autoencoding. The variational autoencoder (VAE) is a method to translate the variational inference process to a deep learning setting. VAEs form the basis of many model-based reinforcement learning approaches (Johnson et al., 2016; Moerland et al., 2017; Buesing et al., 2018; Cornell et al., 2018; Racanière and Weber, 2018), and are used to introduce stochasticity in model dynamics in a scalable way. A notable paper utilizing VAE-based dynamics models is the World Models paper by Ha and Schmidhuber (2018), in which a mixture density model is learned for the car racing environment. In Hafner et al. (2019), the policy component typically encountered in reinforcement learning is swapped for a planning component. Their model learns not only the dynamics but also an estimate of the reward associated with every possible belief state. This allows for the use of the cross entropy method (Rubinstein and Kroese, 2004) to plan trajectories in latent space. In follow-up work (Hafner et al., 2020) the generative model is also used to generate new training data, improving the sample efficiency of the algorithm. Despite using a generative model, these approaches still rely on a scalar reward signal as utility function, whereas the free energy objective combines exploration and exploitation.

The article "Learning Generative State Space Models for Active Inference" was published in 2020. Journal: Front Comput Neurosci.

Ours is not the only work on the intersection between deep artificial neural networks and active inference. In Ueltzhöffer (2018), a generative model for active inference on the mountain car environment was learned using evolution strategies (Salimans et al., 2017) as a policy gradient estimator, while partially fixing the model's state space to allow for easy preferred state specification. More recently in Millidge (2020) the free energy objective is used to learn amortized policies using policy gradient methods on several RL benchmarks. Finally in Tschantz et al. (2019), the application of Bayesian neural networks to model the inherent stochasticity necessary for active inference is explored. However, these applications were still limited to simulated scenarios with low dimensional observations, whereas we learn complex models directly from real-world pixel data.

## 5. Conclusion

In conclusion, we have presented a fully learned way to perform active inference without any prior specification of the agent's belief space. We achieve this by training three different artificial neural networks, each calculating a probability distribution, while minimizing the variational free energy. This way we are able to accurately capture world dynamics, allowing for successful active inference based action selection. We propose a method to estimate the expected free energy from sampled trajectories, effectively implementing active inference as a tree search over policies.

We have demonstrated our approach on three tasks of increasing difficulty. To our knowledge we are the first to successfully apply active inference on real-world, pixel-based inputs without any explicit state space dynamics specification. Our approach makes use of tried and tested deep learning techniques, and is capable of scaling over input and dataset size.

Our current approach relies on the presence of a pre-recorded dataset of (observation, action) pairs. In future work we will focus on learning the model in an online fashion, so that acting and learning can be interleaved, removing the need for a pre-recorded dataset.

## Data Availability Statement

The raw data supporting the conclusions of this article will be made available by the authors, without undue reservation.

## Author Contributions

OÇ and TV conceived and performed the experiments. OÇ, SW, CD, and TV worked out the mathematical basis for the experiments. OÇ, SW, CD, TV, and BD contributed to the paper. Bart supervised the experiments. All authors contributed to the article and approved the submitted version.

The article "Learning Generative State Space Models for Active Inference" was published in 2020. Journal: Front Comput Neurosci.

## Conflict of Interest

The authors declare that the research was conducted in the absence of any commercial or financial relationships that could be construed as a potential conflict of interest.

## Footnotes

^1^A movie demonstrating the results is available at https://tinyurl.com/smvyk53.

## A. Neural Network architectures

**Table A1:** Neural network architectures for the car racing (C.R) and robotic navigation (Robo) experiment.

	**Layer**	**C.R. neurons/filters**	**Robo. neurons/filters**
Posterior	Convolutional	8	8
	Convolutional	16	16
	Convolutional	32	32
	Convolutional	64	64
	Convolutional	128	128
	Concat		
	Linear	128	2 × 128
	Linear	2 × 16	
Likelihood	Linear	16 × 8 × 8	128 × 8 × 8
	Convolutional	128	128
	Convolutional	64	64
	Convolutional	32	32
	Convolutional	16	16
	Convolutional	8	8
	Convolutional	3	3
Trans.	Linear	2 × 16 states	
	LSTM cell		400
	Linear		2 × 128 states

*The convolutional layers in the Likelihood model have a stride and padding of 1 to ensure that they preserve the input shape. All convolutional filters are 3 × 3. Upsampling is done by nearest neighbor interpolation in the Likelihood model after each convolutional layer. The concat step concatenates the flattened processed image pipeline with the vector inputs **a** and **s**. All layers have a leaky ReLU activation function, except for the concat step, which has no activation. For the variance output of the variational layers (denoted with 2x) is activated with a softplus function instead of a leaky ReLU*.
